The article "Emodin enhances osteogenesis and inhibits adipogenesis" was retracted in 2025. Reasons: duplicated images; overlap with earlier publications; unreliable results or conclusions; concerns about the images.

# Emodin enhances osteogenesis and inhibits adipogenesis

**DOI:** 10.1186/1472-6882-14-74

**Published:** 2014-02-24

**Authors:** Feng Yang, Pu-wei Yuan, Yang-Quan Hao, Zheng-Mao Lu

**Affiliations:** 1 Institute of Orthopedics, Shaanxi University of Traditional Chinese Medicine, Century Ave., Xi’an 712000, PR China; 2 Department of Orthopedics, Affiliated Hospital of Shaanxi University of Traditional Chinese Medicine, Xi’an 712083, PR China

**Keywords:** Emodin, Osteogenesis, Adipogenesis, Mesenchymal stem cell, Molecular mechanism

## Abstract

**Background:**

It has been suggested that the formation of osteoblasts in bone marrow is closely associated with adipogenesis, and the balance between osteogenesis and adipogenesis differentiation of MSCs (mesenchymal stem cells) is disrupted in osteoporosis. In order to improve the treatment of osteoporosis, available agents with roles of regulating the balance is highly desirable. Emodin is a natural anthraquinone derivative extracted from Chinese herbs, which have been used to treat bone diseases for thousands of years. However, the underlying molecular mechanisms of emodin in modulating osteogenesis and adipogenesis remain poorly understood.

**Methods:**

The molecular mechanisms of emodin on the processes of osteogenesis and adipogenesis in ovariectomized mouse and BMSCs (bone marrow mesenchymal stem cells) have been studied. We have analyzed the effects of emodin in vivo and in vitro. Female ICR mice were assigned to three groups: sham group, ovariectomy group, emodin group. Efficacy was evaluated by H&E, immunohistochemical assay and Micro-CT. In vitro, we analyze the effect of emodin—at concentrations between 0.1 μM and 10 μM-on the processes of inducing osteogenesis and inhibiting adipogenesis in BMSCs by ALP, Oil red O staining, real time RT-PCR and western blot.

**Results:**

As our experiment shows that emodin could increase the number of osteoblast, BMD (bone mineral density), BV/TV (trabecular bone volume fraction), Tb.N (trabecular number) and Conn.D (connectivity density) of OVX (ovariectomized) mice and decrease the bone marrow fat tissue and adipocytes. The genes and proteins expression of osteogenesis markers, such as Runx2, osterix, collagen type I, osteocalcin, or ALP were up-regulated. While, the genes and proteins involved in adipogenesis, PPARγ, C/EBPα and ap2 were down-regulated.

**Conclusion:**

It proves that emodin inhibits adipocyte differentiation and enhances osteoblast differentiation from BMSCs.

## Background

The decrease in osteoblastogenesis associated with an increasing bone marrow adipogenesis which accompanies osteoporosis in aging populations have long been reported [1,2]. Since osteoblasts and adipocytes are derived from a common multipotential MSC progenitor, it has been proposed that the balance between osteogenesis and adipogenesis differentiation of mesenchymal stem cells (MSCs) is disrupted in osteoporosis [3]. The consequence of these changes is a progressive marrow adiposity that accompanies osteoporosis in the aging process. Several agents, including drugs, oxidative stress, nutrients, hormones, and metabolic signals, can switch multipotent MSC differentiation toward adipocyte or osteoblast formation [4]. Regulator in the balance between osteogenesis and adipogenesis of MSCs may be a novel therapeutic target.

Emodin, (1, 3, 8-trihydroxy-6-methylan-thraquinone, molecular structure is Figure 1) a natural anthraquinone derivative found in the roots and rhizomes of numerous plants such as Polygonum multiflorum, rhubarb, Alose. has been demonstrated to possess multiple biological activities and abilities to ameliorate metabolic disorders [5]. In addition, hydroxyanthraquinones such as emodin, are phytoestrogens with an affinity to human estrogen receptors [6]. Polygonum multiflorum which active component is emodin, has been used to treat osteoporosis in traditional Chinese medicine for a long time. Pharmacological studies have demonstrated that emodin exhibits anti-cancer, anti-inflammatory, anti-fibrosis effects [7-9]. The research on anti-bone loss and anti-adipogenesis is a few. Lee SU et al. reported that emodin could activate the mRNA expression of bone morphogenetic protein (BMP)-2 in the mouse osteoblast [10]. Emodin has effect on the inhibition of mouse 3 T3-L1cell’s proliferation and differentiation [11]. Yang’s data suggest emodin could inhibit the proliferation and differentiation of preadipo -cytes in a dose and time dependent manner, and induce apoptosis of preadipocytes in a certain degree [12]. This kind of studies showed that the emodin promoted osteoblastic differentiation and inhibited adipocytic differentiation. The limitation of previous studies is that they did not evaluate the effect of emodin at the tissue level and on BMSC differentiation. Therefore, the effect of emodin on the balance of osteogenesis and adipogenesis has been investigated both in vitro and in vivo. A novel therapeutic target of emodin for osteoporosis have been found.

**Figure 1:** **The structure of emodin. (A)** Molecular formula: C_15_H_10_O_5_, molecular weight: 270.23. HE Staining showed more osteoblasts attaching to the surface of bone trabeculae of emodin-OVX group **(C)** and SHAM group **(B)** than OVX group **(D)**. Osteoblast activity scores from HE staining slices: N.ob/T.Ar (osteoblast number per trabecular area). **(E)** and N.ob/B.PM (osteoblast number per bone perimeter) **(F)** rose up in OVX + emodin group. The columns represent the mean ± SE of three independent experiments. *: P < 0.05 vs. OVX. Immunohistochemical assessments of the protein of Runx2 **(G, H, I)** and PPARγ **(J, K, L)**. Immunohistochemical analysis showed more increase in Runx2 protein distribution in the OVX + emodin groups than OVX group. Immunohistochemical analysis showed more increase in PPARγprotein distribution in the OVX + emodin groups. Representative 3-D images of lumbar vertebral body of sham-operated mice (**M**:SHAM), ovariectomy mice (**N**:OVX) and emodin-treated OVX mice (**O**:OVX + emodin) by micro-CT. Bone loss and trabecular bone deterioration are evident in the OVX group and the progression of bone loss and bone deterioration is partially rescued by emodin treatment.

## Methods

### Animal grouping and treatments

Thirty 6-month-old ICR female mice were purchased from Shanghai Laboratory animal center (SCXK2007-0005). The study was conducted in the Institute of Orthopedics, Shaanxi University of Traditional Chinese Medicine. The animal handlings and experimental procedures were approved by the Committee on the Ethics of Animal Experiments of Shaanxi University of Traditional Chinese Medicine, which conforms to the Guide for the Care and Use of Laboratory Animals published by the US National Institutes of Health.

The mice were divided into three groups: (1) Sham-ovariectomized group (sham), (2) ovariectomized group (OVX), (3) ovariectomized group treated with emodin (OVX + E). Mice were anesthetized with ketamine and were positioned dorsal side up. Aseptically, each fallopian tube was located bilaterally and both ovaries were removed. The transection sites were ligated. Each surgical procedure is same, the mice in OVX + E group were intraperitoneal injected with emodin at dose of 100 mg/(kg · d) twice every three days for three months after the OVX surgery.

### Histomorphology evaluation

Lumbar vertebra was prepared for the bone histomorphology analysis. Decalficied frontal sections of lumbar vertebra were embedded in paraffin wax and cut (6 μm thickness) using a microtome (Leica EG1160, Germany). The histological section was stained by haematoxylin & eosin (H&E). Sections were examined by using a photomicroscope set (Olympus DP71; Olympus, Tokyo), and morphometric study was performed by using an image processing and analysis software (Mediacybernetics, USA).

Moreover, Bone marrow was taken from the anterior iliac crest with needle. Plastic embedding of undecalcified cores was used. Sections 3 μm in thickness were stained with Gill’s hematoxilin. From each specimen, 8 to 10 random microphotographs were obtained for the Image Pro Plus 6.0 software analysis. In each specimen, the following morphometric parameters were determined: (1) percent of marrow fat tissue fraction; (2) number of adipocytes/mm^3^.

### Immunohistochemical staining for Runx2 and PPARγ

Immunohistochemical staining was performed in 6 μm-thick paraffin sections mounted on positive-charged slides. Sections were deparaffinized with xylene and rehydrated through descending concentrations of ethanol. Antigen retrieval was performed by heating the slides in Target Retrieval Solution, pH 9.0 (Dako Denmark, Glostrup, Denmark) at 97°C in a water quench for 5 min for the interstitial and cell surface antibodies or with boiling citrate buffer, pH 6.0 for 20 min in a microwave oven for nuclear markers.

The following primary antibodies were applied overnight at 4°C: rabbit polyclonal anti- Runx2 (1:50 dilution; Abcam), and rabbit polyclonal anti-PPARγ (1:50 dilution; Abcam). Biotinylated secondary antibody (anti-rabbit, BioGenex) was applied for 20 min at 37°C, and then the slides were exposed to a streptavidin-biotin, alkaline phosphatase complex. Negative controls were performed by omitting the primary antibody. The color reaction was elicited by using 3, 3′-diaminobenzidine (DAB) solution (invitrogen, USA), visualized, and examined by using a photomicroscope set (Olympus DP71).

### Bone microarchitecture assessment by microcomputed tomography

Bone microarchitecture in lumbar vertebra was assessed using microcomputed tomography (μCT) (MicroCT80, SCANCO Medical, Switzerland). Trabecular bone of the lumbar vertebra was scanned so that 250 images were acquired. All scans were performed in a 1,024 × 1,024 matrix resulting in an isotropic voxel resolution of 16 μm in all three spatial dimensions. An integration time of 150 ms per projection was used.

The scanning procedure and reconstruction of 3-D images were performed. Trabecular parameters included trabecular bone volume fraction (BV/TV, percent), number (Tb.N, number per millimeter), thickness (Tb.Th, micrometer), and separation (Tb.Sp, micrometer).

### Osteoblast and adipocyte differentiation

BMSCs were obtain from the bone marrow of the bilateral tibia and femur of eight mice per group. The cells were thawed and seeded in α-minimum essential medium (α-MEM, Gibco, invitrogen, USA), 10% fetal bovine serum (FBS, Gibco, invitrogen, USA), Grown and confluent cells were trypsinized, collected, and plated at 500 cells per square centimeter in 100 mm plates (Corning incorporated, USA). When the cells came closer to confluence, the differentiation was initiated by means of specific media. The osteoblast media (OM) also contained 10^−8^ M dexamethasone, 10 mM β-glycerophosphate, and 0.05 mM L-ascorbic acid, while the adipocyte media (AM) contained 10^−6^ M dexamethasone, 0.5 mM isobutylmethylxanthine, 100 μM indomethacin and insulin 10 mg/L. Treatment with emodin (purity >80%; molecular weight: 270.23; purchased from You-si Biotech Co. Shanghai, China) started at the same time as the differentiation process. The toxicity of these concentrations of emodin on the MSCs was tested by MTT assay. Logarithmic phase cells were collected and seeded in 96-wells plate at a density of 1000-10000/well at 37°C, After the cells attached, different concentration of emodin were added to the medium and incubated 16-48 hours. MTT (5 mg/ml) was dissolved in PBS. 20 μl of MTT solution was added to each well and incubate at 37°C for 4 hours. The medium was removed with syringe. 150 μl of DMSO was added to each well and pipette up and down to dissolve crytals. The plate was measured absorbance at wavelength at 570 nm.

### Real time PCR

Total RNA was obtained from cells in culture using Trizol Reagent (Invitrogen, USA), according to the manufacturer’s instructions, and cDNA was synthesized from total RNA (iScript™ cDNA Synthesis Kit, Bio-Rad), which had been previously treated with DNAse I (Sigma-Aldrich) following the manufacturer’s instructions. Real-time polymerase chain reaction (RT-PCR) to quantify the mRNA of osteoblastic and adipocytic markers was performed in the Rotor-Gene 3000 (Corbett Research, Australia) using SYBR® Green as a double-strand DNA-specific binding dye. PCR reactions were carried out in a final volume of 20 μl, with 1 μl of cDNA sample, 1 μl of each primer (Table 1), and Quantitect® SYBR® Green master mix (TaKaRa BIO). The conditions for the Rotor-Gene 3000 were 95°C for 15 min, 40 cycles of 95°C for 30 s, 60°C for15 s, and 72°C for 30 s. The relative expression of mRNA was calculated according to the 2^-ΔΔCt^ method. The endogenous control is β-actin.

**Table 1:** Mouse primers for real-time quantitative PCR assays

**Genes**	**Forward primer**	**Reverse primer**
β-actin	5′-CTTAGTTGCGTTACACCCTTTCTTG-3′	5′-CTGCTGTCACCTTCACCGTT CC-3′
ALP	5′-CATGAAATACGAGATCCACCGAGAC-3′	5′-ATGCGACCACC CTC CACGAAG-3′
Runx2	5′-CATGGTGGAGATCATCGC-3′	5′-ACT CTT GCC TCG TCC ACT C-3′
Osterix	5′-GCA GCTAGAAGGGCGTGGTG-3′	5′-GCAGGCAGGTGAACTTCTTC-3′
OC	5′-GAGGGCAGCGAGGTAGTGAAG-3′	5′-GATGTGGTCAGCCAACTCGTCA-3′
ColI	5′-TCCGACCTCTCTCCTCTGAA-3′	5′-GAGTGG GGTTATGGAGGGAT-3′
BMP4	5′-TGAGCCTTTCCAGCAAGTTT-3′	5′-CTTCCCCGTCTCAGGTATCA-3′
PPARγ	5′-CCAGAAAGCGATTCCTTCAC-3′	5′- CACGTTAGTTTCACCTCGGA-3′
C/EBPα	5′-AAGAAGTCGGTGGACAAGAACAG-3′	5′-TGCGCACCGCGATGT-3′
ap2	5′-GGCCAGGAATTTGACGAAGTC-3′	5′-AGCGTAACTTGAGATGTTGTAAGACA-3′

### ALP staining

To confirm osteogenesis, cells cultured in osteogenic media (OM) were stained using 1-step NBT/BCIP (Thermo scientific). The cells were fixed in 4% paraformaldehyde for 10 min, washed with dH_2_O, mixed the 1-step NBT/BCIP until desired stain developed.

### Oil red O staining

To confirm adipogenesis, cells cultured in adipogenic media (AM) were stained using oil red O (Sigma). The cells were fixed in 4% paraformaldehyde for 10 min, washed with dH_2_O, and incubated with an oil red O solution for 20 min at room temperature (RT). Then the cells were rinsed with dH_2_O, counterstained with Gill’s Hematoxylin II (Sigma-Aldrich), and viewed under a light microscope.

### Western blot analysis

To examine the effect of emodin on Runx2 and PPARγ protein, primary BMSCs were seeded in 6-well plates at a density of 5 × 10^6^ cells/well. Culture cells were treated with emodin for 21 days. Cells lysates were extracted with RIPA protein extraction reagents (Beyotime) according to the manufacturer’s protocol. Proteins were transblotted onto a PVDF membrane (BIO-RAD) and the membrane was blocked with 5% milk in PBST for 1 hour at room temperature (RT). The samples were incubated with the primary antibody overnight at 4°C and the HRP-conjugated secondary antibodies (Abcam) for 1 hour. The polyclonal rabbit Runx2 antibody and the polyclonal rabbit PPARγ antibody were obtained from Abcam. After the immunocomplex was removed by stripping buffer (Chemicon Int.), the same membrane was reblotted with mouse anti-β-Actin antibody (Sigma) for the loading control. Then visualized with Odyssey infrared imaging system (Li-COR inc.) according to the manufacturer’s instructions.

### Statistical analysis

All the assays were made twice. The data are expressed as the average with its SE. The statistical analysis was carried out using the SPSS 17.0 software. The results obtained from these two independent experiments were compared using the one-way ANOVA followed Tukey’s test, and the differences were considered significant when p < 0.05.

## Results

### Histomorphology analysis

It revealed that cancellous bone was formed of a dense network of bone trabeculae in the SHAM group and osteocytes appeared in their lacunae (Figure 1B). The endosteal surface of trabeculae was lined by osteoprogenitor cells, osteoblasts and osteoclasts in Howship’s lacunae. Bone marrow spaces were seen between the trabeculae.The results in the OVX-mice revealed the cancellous bone trabeculae lost their normal architecture and appeared discontinuous and thinning. While bone marrow spaces widened (Figure 1C). Osteoclasts were apparently increased as compared with the sham group. Erosion cavities were detected in the endosteal surface in some trabeculae and proliferation of osteoblasts was also detected in some areas.The emodin-OVX mice showed marked improvement as compared to the OVX-mice. The cancellous bone trabeculae partially regained near normal structure and the trabecular bone widened, its broken points lessened and its Howship’s lacunae shallowed as compared to the SHAM- operated control group (Figure 1D).Meanwhile, quantitation showed that the number of osteoblasts was increased at unit tissue area and unit bone perimeter in the OVX and emodin-OVX group (P < 0.05), the osteoblast number in sham group was non-significant different from that in the emodin- OVX group (Figure 1E, F).

To evaluate the effect on bone marrow fat tissue and adipocytes, the values of two parameters (fat tissue fraction and number of adipocytes/mm^3^) were significantly higher in OVX as compared with sham and emodin (Table 2). The difference between the emodin and OVX group was significant. The data indicates emodin can decrease the bone marrow fat tissue and adipocytes of OVX mice.

**Table 2:** Effect of emodin on fat tissue and adipocytes in bone marrow

**Group**	**Fat tissue fraction (%)**	**Number of adipocytes/mm**^**3**^
Sham	18.40 ± 1.51	2040.05 ± 358.65
OVX	41.39 ± 2.60	4219.18 ± 432.30
Emodin	22.52 ± 3.48*	2627.08 ± 467.09*

Data are presented as mean ± SEM *significantly different from the OVX group:P < 0.05.

### Immunohistochemical staining for Runx2 and PPARγ

Immunohistochemical study of the section in the OVX-mice revealed strong immunoreactivity for PPARγ, while much weaker immunostaining for Runx2. However, the density of the Runx2 positive staining of the Emodin-OVX group increased dramatically compared with the OVX group (Figure 1G, H, I). And immunohistochemical staining for PPARγ was weaker after emodin treatment (Figure 1J, K, L).

### Bone microarchitecture assessment by microcomputed tomography

There was a significant difference in trabecular parameters between the OVX group and emodin-OVX group (Table 3). 3-D images showed deterioration of trabecular bone morphology in the ovariectomized mice. Bone trabecular appeared discontinuous and lessen. while these progression of bone loss and deterioration is partially rescued by emodin in emodin-OVX mice (Figure 1L, M, N).

**Table 3:** Effect of emodin on trabecular bone microarchitecture

	**BMD**	**BV/TV**	**Tb.N (1/mm)**	**Tb.Th (mm)**	**Tb.Sp (mm)**	**Conn.D (1/mm**^**3**^**)**
Sham	2.93 ± 0.07	0.25 ± 0.02	3.75 ± 0.13	0.12 ± 0.03	0.31 ± 0.06	115 ± 3.28
OVX	1.57 ± 0.11*	0.15 ± 0.02*	2.42 ± 0.16*	0.06 ± 0.02*	0.54 ± 0.08*	76 ± 2.32*
Emodin	2.85 ± 0.06**	0.22 ± 0.01**	3.28 ± 0.18**	0.09 ± 0.02	0.41 ± 0.05**	96 ± 2.76**

Data are presented as mean ± SEM (n = 8) *significantly different from the sham group:P < 0.05. **significantly different from OVX group: P < 0.05.

### Emodin enhanced BMSC proliferation

Structure of emodin was shown in Figure 1A. The effect of emodin on cell proliferation of BMSC has been tested by MTT assay. As shown in Figure 2A, emodin has significant effects on cell growth at the concentrations of 0.1 μM-10 μM after 3-d treatment, and emodin show inhibition on cell proliferation at 2d. However, when the dose reached 100 μM, Emodin started to show toxic effect. Based on these observations, 0.1 μM, 1 μM and 10 μM of emodin were used in the following experiments.

**Figure 2:** **Emodin can stimulate cell proliferation.** It stimulates osteogenesis differentiation of BMSC. When it (0.1-10 μM) was added to the OM culture of BMSC for 7, 14, 21 days. Quantitative PCR (qPCR) assay was performed to examine the expression of osteogenesis-specific genes. **A)** MTT assays showed that emodin have significant effects on cell growth at the concentrations used (0.1-10 μM), but there are inhibition at 100 μM after 3 days treatment in BMSC (*p* > 0.05, compared with the group without emodin). In addition, emodin at concentrations of 0-100 μM are inhibition at 48 h. **B)** Emodin increased the mRNA expression of BMP4 in BMSC in a dose-dependent manner, with more pronounced effect at the concentration of 10 μM. **C)** Treatment with emodin at the concentration of 10 μM also significantly increased the mRNA expression of Runx2 in osteogenesis differentiation of BMSC for 14 days and 21 days. **D)** Emodin increased the osterix mRNA expression. **E)** Emodin dose-dependently enhanced the alkaline phosphatase (ALP) activity in BMSC, especially at the concentration of 10 μM. **F**) Emodin dose-dependently enhanced the ColI mRNA expression. **G)** Emodin increased OCmRNA expression at concentrations of 10 μM for 21 days. **H)** Western blotting analyses of the protein abundance of Runx2. β-actin was used as an invariant control for equal loading. P < 0.05 vs OVX group. ALP staining **(I**, **J**, **K** and **L)** also showed treatment with emodin at the concentrations of 0.1and 10 μM increased the ALP activity in BMSC compared with the group without emodin.

### Emodin up-regulates mRNA and protein expression of osteogenesis markers

Changes in gene expression, as well as in the osteoblast phenotype, were observed when emodin was present in the OM. The expression of BMP_4_ genes induced by OM with emodin was increased in compared with the cells not treated with emodin (Figure 2B). After 14 days of differentiation and treatment, this increase was higher when the concentration of emodin was 10 μM in the gene studied, and this great increase continued for 21 days. The expression of transcription factors Runx2 and osterix were influenced positively. The expression of Runx2 was significantly higher in treated cells than in induced but nontreated cells after 21 days (Figure 2C). But the increase of osterix expression was only shown after 21 days of treatment (Figure 2D). In addition, the presence of emodin in the OM produced an increase in the expression of the ALP gene (Figure 2E), especially, at the concentration of 0.1 μM in 7 days.Moreover, the expression of genes involved in the formation of the cellular matrix was also increased by the presence of emodin. On the seventh day of treatment, the levels of expression for collagen type I were higher when the concentrations were 1 μM or 10 μM (Figure 2F). After 14 days, a significant increase in collagen expression was observed at a concentration of 10 μM and in osteocalcin expression at 1 μM of emodin (Figure 2G). In addition, emodin significantly increased Runx2 protein expression by western blot analysis (Figure 2H).The influence of emodin on the development of the osteoblast phenotype from MSCs was evaluated by monitoring the formation. When emodin was added to the OM medium, the phosphatase alkaline staining showed an increase in comparison with cells not treated with emodin (Figure 2I, J, K, L).

### Emodin down-regulates mRNA and protein expression of adipogenesis markers

The expression of three marker genes for adipogenesis—the transcription factor peroxisome proliferator-activated receptor gamma (PPARγ), C/EBPα and the fatty acid-binding protein (ap2) gene—was studied in order to analyze the effect of emodin on the differentiation of MSCs into adipocytes.The expression of PPARγ was inhibited at the first moment of differentiation and treatment with the three concentrations of emodin. The rate of inhibition was inversely proportional to the emodin concentration, and maximum inhibition across the three concentrations was seen at 21 days (Figure 3A). The C/EBPα expression was inhibited by emodin (Figure 3B); however, in the case of 10 − 4 M, this inhibition was not observed until 14 days of differentiation and treatment. Moreover, the ap2 expression was also inhibited in other cellular cultures differentiated with AM plus emodin (Figure 3C). Emodin significantly decreased PPARγ protein expression by western blot analysis (Figure 3D).In addition, the influence of emodin on the adipocyte phenotype was evaluated. The formation of lipid droplets, a characteristic of the adipocyte formation process, was monitored using the oil red O staining. There were major changes in the phenotype of differentiating MSCs in the treated cells, mainly a decrease in the development and accumulation of fat in the cells. So, the area occupied by the lipid droplets was reduced at the three concentrations of emodin and at all the time points, differentiations were analyzed (Figure 3E). Aside from this, there was no difference in fat accumulation due to the concentration of emodin. And the size of the fat particles was smaller compared with nontreated cells at 21 days of differentiation and treatment (Figure 3F, G, H, I).

**Figure 3:** **Emodin inhibits adipogenesis differentiation of BMSC.** It (0.1-10 μM) was added to the AM culture of BMSC for 7, 14, 21 days. Quantitative PCR (qPCR) assay was performed to examine the expression of adipogenesis-specific genes after treatment with emodin. **A)** Emodin decreased the expression of PPARγmRNA in BMSC in a dose-dependent manner, with more pronounced effect at the concentration of 10 μM. **B)** Treatment with emodin at the concentration of 10 μM also significantly decreased the expression of C/EBPαmRNA in osteogenesis differentiation of BMSC for 14 days and 21 days. **C)** Emodin dose-dependently enhanced the ap2 in adipogenesis differentiation of BMSC, especially at the concentration of 10 μM. **D)** Western blotting analyses of the protein abundance of PPARγ. β-actin was used as an invariant control for equal loading. P < 0.05 vs OVX group. **E)** The number of lipid droplets that was formed from the BMSCs of emodin-OVX was significantly lower than that formed from the BMSCs of OVX. Data are presented as mean ± SEM. Data presented are three independent experiments with triplicates within each experiment. P < 0.05, significantly different from the OVX group. Oil red O staining also showed treatment with emodin at the concentrations of 0.1 μM and 10 μM inhibited the adipogenesis differentiation of BMSC. *p < 0.05, when compared with the group without emodin **(F, G, H, I)**.

## Discussion

It has been proposed that the close relationship between increased adipocytes and decreased bone formation in conditions of bone loss like age-related osteoporosis [13,14].

There are some evidences for a reciprocal relationship between these cell lineages [15,16].

It has been suggested that targeting regulatory factors that alter mesenchymal cell fate to increase the number of osteoblasts and decrease adipocytes have the potential to provide novel therapeutic approaches for osteoporosis.

This study provides the evidence for the therapy of herbs containing emodin for osteoporosis, and reveals the effect of emodin on enhancing osteogenesis and inhibiting adipogenesis in vitro and in vivo. The emodin prevents bone loss by modulating the differentiation of the osteogenic and adipogenic lineages, as shown in the enhancement of the osteogenic gene expression markers and osteoblast phenotypic characteristics, eventually promoting osteoblastogenesis. We hypothesize that emodin might protect the bone from bone volume loss by enhancing osteogenesis and inhibiting adipogenesis differentiation of BMSC. This prompted us to determine the histomorphometric parameters of trabecular bone after treating OVX-induced osteoporotic mice with emodin. It proved osteoblast number of emodin-OVX group was higher than OVX group.

The values of trabecular bone volume, trabecular number and connectivity density in the emodin-treated OVX mice were higher than those determined in OVX mice.

The result of immunohistochemical staining suggests that emodin increases the protein level of Runx2 and decreases that of PPARγ. This result suggests that emodin exert a balance between bone formation and bone marrow fat at the tissue level.

To explore the cellular and molecular mechanisms of the anabolic action of emodin on bone formation and inhibiting bone marrow fat, the present study assessed the capacity of osteogenesis and adipogenesis differentiation of BMSCs. Runx2 is a master transcription factor regulating both embryonic bone development and postnatal osteoblastic function [17]. Increments in Runx2 expression stimulate mesenchymal cells to differentiate into osteoblasts [18]. Osx acts downstream of Runx2/Cbfa1 [19]. Both are involved in the cellular decision to initiate differentiation into an osteoblast and play a critical role in maintaining osteoblast-specific expression during osteoblastgenesis [20]. Similarly, the important role of emodin in osteoblast differentiation is also supported by the observation of higher levels of expression of other osteoblast markers, such as ALP gene expression and activity or the type I collagen gene expression. On protein level, emodin increase Runx2 protein expression. Our results further demonstrate that emodin in the AM caused a decrease in adipocyte formation from MSCs. The expression of the most important regulators of adipogenesis, the PPARγ, was inhibited in mRNA and protein by emodin. Moreover, the expression of the other adipogenic marker genes, such as ap2 and C/EBPα, and the phenotypic characteristic of adipocytes, as fat accumulators, showed a decrease when emodin was present.

Recent advances in the elucidation of the pathophysiology of osteoporosis in the elderly indicate that the loss of balance between osteoblastogenesis and adipogenesis in bone marrow cell differentiation is a key mechanism of osteoporosis in older adults [21]. Indeed, in ovariectomized rats, bone fat increases in parallel with bone loss [22]. Adipocyte differentiation is under the control of PPARs, members of the nuclear receptor superfamily, in concert with members of the C/EBP family of basic leucine zipper nuclear transcription factors [23]. Previous studies have demonstrated the PPARγ ligands have the potential to inhibit β-catenin signaling [24] and inhibit Runx2-mediate transcription of osteogenesis-related genes [25]. Our findings show that emodin reduces the expression of PPARγ, inhibits adipocyte differentiation, and enhances differentiation into osteoblast. When PPARγ gene up-regulats, the Runx2 and osterix inhibits. Therefore, this upward regulation of osteogenesis gene expression by emodin could be the mechanism through which this anthraquinone derivative drives its osteogenesis differentiaton and inhibited adipogenesis differentiation on MSC. In this way, emodin may be an antagonizes of the potential actions of the exogenous ligands of PPARγ. In addition, in spite of the limitations in this study, these data can explain in part that the Chinese herbs containing emodin could contribute to decreasing the risk of developing osteoporosis.

## Conclusion

Taken together, the present data demonstrated that emodin treatment exerted its anabolic effects on trabecular bone in an ovariectomized mice model of osteoporosis by increasing bone formation and decreasing bone marrow fat. These data in vitro suggest that the emodin can regulates the balance of MSCs differentiation into osteoblasts and adipocytes. Therefore, further studies should be pursued to test this effect in clinical trials to determine whether emodin could be used as a drug or nutrient.

## Abbreviations

MSCs: Mesenchymal stem cells; BMSC: Bone marrow mesenchymal stem cells; BMD: Bone mineral density; OVX: Ovariectomized; Runx2: Runt-related transcription factor 2; PPARγ: The peroxisome proliferator-activated receptor gamma; C/EBPα: CCAAT- enhancer binding protein; ap2: Fatty acid binding protein; AM: Adipocyte media; OM: Osteoblast media.

## Competing interest

All authors have no conflicts of interest.

## Authors’ contributions

FY contributed to the design of the study. PWY, YQH and ZML contributed to the creation of the Manual of Procedures, implementation of the study protocol and acquisition of data. FY drafted the manuscript, and all authors provided critical revision and have approved the final manuscript.

## Pre-publication history

The pre-publication history for this paper can be accessed here:

http://www.biomedcentral.com/1472-6882/14/74/prepub
